The article "Effects of drought stress on global gene expression profile in leaf and root samples of Dongxiang wild rice (Oryza rufipogon)" was published in 2017. Journal: Biosci Rep.

# Effects of drought stress on global gene expression profile in leaf and root samples of Dongxiang wild rice (*Oryza rufipogon*)

**DOI:** 10.1042/BSR20160509

**Published:** 2017-06-27

**Authors:** Fantao Zhang, Yi Zhou, Meng Zhang, Xiangdong Luo, Jiankun Xie

**Affiliations:** Plant Functional Genomics Laboratory, College of Life Sciences, Jiangxi Normal University, Nanchang, 330022, China

**Keywords:** Drought-stress resistance, genetic resources, Illumina sequencing, transcriptome, wild rice

## Abstract

Drought is a serious constraint to rice production throughout the world, and although Dongxiang wild rice (*Oryza rufipogon*, DXWR) possesses a high degree of drought resistance, the underlying mechanisms of this trait remains unclear. In the present study, cDNA libraries were constructed from the leaf and root tissues of drought-stressed and untreated DXWR seedlings, and transcriptome sequencing was performed with the goal of elucidating the molecular mechanisms involved in drought-stress response. The results indicated that 11231 transcripts were differentially expressed in the leaves (4040 up-regulated and 7191 down-regulated) and 7025 transcripts were differentially expressed in the roots (3097 up-regulated and 3928 down-regulated). Among these differentially expressed genes (DEGs), the detection of many transcriptional factors and functional genes demonstrated that multiple regulatory pathways were involved in drought resistance. Meanwhile, the DEGs were also annotated with gene ontology (GO) terms and key pathways via functional classification and Kyoto Encyclopedia of Gene and Genomes (KEGG) pathway mapping, respectively. A set of the most interesting candidate genes was then identified by combining the DEGs with previously identified drought-resistant quantitative trait loci (QTL). The present work provides abundant genomic information for functional dissection of the drought resistance of DXWR, and findings will further help the current understanding of the biological regulatory mechanisms of drought resistance in plants and facilitate the breeding of new drought-resistant rice cultivars.

## Introduction

Drought, which remains one of the most important natural hazards facing our world today, affects agricultural productivity and can potentially reduce global crop yield by up to 20% annually [1,2]. Among the world’s most important food crops, rice (*Oryza sativa*) serves as the staple food for more than half the world’s population, and as a typical semiaquatic plant, the crop is able to grow well in waterlogged soil [3]. However, rice is highly sensitive to drought, and when rice plants are exposed to drought stress, they respond by activating a series of complicated regulatory mechanisms [4].

The article "Effects of drought stress on global gene expression profile in leaf and root samples of Dongxiang wild rice (Oryza rufipogon)" was published in 2017. Journal: Biosci Rep.

In rice, drought resistance is a complex trait that is regulated by polygenes or gene complexes, and recent advances in molecular biology have facilitated the isolation and identification of increasing numbers of these genes [4,5]. Such genes have been reported to encode a variety of proteins, including transcription factors (TFs), protein kinases, enzymes related to plant hormone synthesis and other regulatory and functional proteins [6–8]. However, the regulatory mechanisms of drought resistance have not been fully understood. Thus, a better understanding of drought-resistance mechanisms would be helpful for breeding drought-resistant rice cultivars, in order to stabilize rice production.

Our previous studies demonstrated that an accession of wild rice (*Oryza rufipogon*) collected from Dongxiang County, Jiangxi Province, China (Dongxiang wild rice, i.e. DXWR) is found in more northern habitats (28º14′ N) than other common wild rice species in China and even in the world [9]. DXWR possesses strong drought resistance, with an ability to survive under extreme drought conditions [10,11]. However, the molecular mechanism and regulatory network of the accession’s drought resistance remain unclear, and to date, only 12 quantitative trait loci (QTLs) related to drought resistance in DXWR have been identified [12].

Gene expression profiling can accelerate the progress toward a comprehensive understanding of the molecular mechanisms that control responses to environmental stress. Recently, high-throughput sequencing technology has been widely applied to investigate drought stress-induced transcription in a variety of plants, including coffee [13], cassava [14], sorghum [15], peanut [16], and maize [17], but the transcription profile of drought-stressed DXWR has yet to be reported.

Therefore, the main objective of the present study was to investigate the expression profiles of drought-stressed DXWR and to uncover candidate genes by combining differentially expressed genes (DEGs) with previously identified drought resistance-related QTL intervals. The results will provide new insights into the molecular mechanism of drought resistance and will accelerate the utilization of genetic resources from DXWR for drought-resistant breeding in rice.

## Materials and methods

### Plant materials, growth conditions, and drought treatment

DXWR is conserved *ex situ* at the Jiangxi Academy of Agricultural Sciences (JXAAS, http://www.jxaas.com/), Nanchang, China, and the seeds of DXWR are freely available for scientific research. In the present study, the plants were grown and the drought treatments performed following the methods described in the previous paper [11]. Briefly, the uniformly germinated seeds of DXWR were grown in a plastic pot in a plant growth chamber at day/night temperature of 30°C/26°C (14 h day/10 h night) with 3000 lux of light intensity and relative humidity of 70%, and with IRRI (International Rice Research Institute) nutrient solution (1.25 mM NH_4_NO_3_, 0.3 mM KH_2_PO_4_, 0.35 mM K_2_SO_4_, 1 mM CaCl_2_.2H_2_O, 1 mM MgSO_4_.7H_2_O, 0.5 mM Na_2_SiO_3_, 20 μM NaFeEDTA, 20 μM H_3_BO_3_, 9 μM MnCl_2_.4H_2_O, 0.32 μM CuSO_4_.5H_2_O, 0.77 μM ZnSO_4_.7H_2_O, and 0.39 μM Na_2_MoO_4_.2H_2_O, pH 5.5) as described previously [18]. At the four-leaf stage, the half of the seedlings were air dried in the growth chamber until the leaves appeared wrinkled for drought-stress treatment, whereas, the other half of the seedlings were allowed to continue growth in the IRRI nutrient solution for control treatment (Supplementary Figure S1). Leaf (leaves with dry treatment (LD)) and root (roots with dry treatment (RD)) tissues from the drought-stressed group and leaf (leaves without dry treatment (LCK)) and root (roots without dry treatment (RCK)) tissues from the control group were collected and immediately frozen in liquid nitrogen. For each group and tissue type, samples were collected from ten plants and mixed, in order to minimize the effect of transcriptome unevenness among plants.

The article "Effects of drought stress on global gene expression profile in leaf and root samples of Dongxiang wild rice (Oryza rufipogon)" was published in 2017. Journal: Biosci Rep.

### RNA extraction, cDNA library preparation, and transcriptome sequencing

Total RNA was extracted using TRIzol reagent (Invitrogen, Carlsbad, CA, U.S.A.), according to the manufacturer’s instructions, and the quality and quantity of the resulting RNA were examined using agarose gel electrophoresis and an ND-1000 spectrophotometer (NanoDrop Technology, Wilmington, DE, U.S.A.). Next, cDNA libraries were constructed from the RNA of the four tissue samples (LD, RD, LCK, and RCK) and sequenced by the Beijing Genomics Institute (BGI, Shenzhen, China). Briefly, mRNA was isolated from the total RNA using magnetic beads and fragmented into short sequences that were used as templates for cDNA synthesis. After end repair, adapter ligation, and PCR amplification, paired-end cDNA libraries were constructed and sequenced using an Illumina HiSeq™ 2000 sequencing platform.

### Reads filtration and functional annotation of unigenes

High-quality clean reads were obtained by removing adapter sequences from the raw reads and by excluding sequences that contained >10% unknown bases and >50% low-quality bases with a *Q*-value <20 [19]. The retained high-quality reads were mapped to the Nipponbare reference genome by TopHat software (-N, 2-read gap length, 3-read edit distance, 3-read realign edit distance, 0-report secondary alignments coverage search, microexon-search library type, fr-unstranded, b2-sensitive) [20,21], and a RABT (Reference Annotation Based Transcript) assembly was generated from the aligned reads using Cufflinks [22]. For functional annotation, all the unigenes were searched against the NCBI Nt (https://www.ncbi.nlm.nih.gov/) and Nr (http://www.ncbi.nlm.nih.gov/) databases, as well as against the Swiss-Prot (http://www.expasy.ch/sprot/), COG (http://www.ncbi.nlm.nih.gov/COG/), and Kyoto encyclopedia of genes and genomes (KEGG) (http://www.genome.jp/kegg/) databases, using the BLASTN or BLASTX algorithms with an E-value cutoff of 10^−5^ [23]. The Blast2GO program was used to assign gene ontology (GO) terms to the unigenes from the leaf and root tissues, using a *P*-value cutoff of 0.05 [24].

The article "Effects of drought stress on global gene expression profile in leaf and root samples of Dongxiang wild rice (Oryza rufipogon)" was published in 2017. Journal: Biosci Rep.

### Identification of differentially expressed unigenes

The expression of each gene was calculated by quantitating the reads according to the RPKM (reads per kilobase per million reads) method [25]. An FDR (false discovery rate) of ≤0.001 and absolute log_2_RPKM ratio of ≥1 were used as significance thresholds for differences in gene expression [26].

### Validation of transcriptome sequencing

To confirm the gene expression data, quantitative real-time PCR (qRT-PCR) was performed on 30 randomly selected DEGs (15 up-regulated and 15 down-regulated). The qRT-PCR was implemented using the SYBR Premix Ex Taq Kit on a Chromo 4 real-time PCR detection system (Bio–Rad, Hercules, CA, U.S.A.) and the primers are listed in Supplementary Table S1. The relative expression values were calculated using the 2^−ΔΔ*C*^_t_ method, with *OsActin1* as the internal control [27]. All reactions were performed using one biological sample and three technical replicates.

## Results and discussion

### Transcriptome sequencing statistics

In total, 46.8, 48.7, 43.6, and 46.7 million high-quality paired-end reads were generated by Illumina sequencing the LCK, LD, RCK, and RD cDNA libraries, respectively (Table 1). Now, it is well-accepted that cultivated rice was domesticated from common wild rice thousands of years ago [28]. Furthermore, Xie et al. [9] revealed that DXWR was genetically closer to *Oryza sativa* ssp. *japonica* than *indica*. The Nipponbare (*O. sativa* ssp. *japonica*) genome has been completely sequenced with Sanger sequencing technology and is ranked as the best assembled and annotated one out of all rice genomes [29,30]. Therefore, in the present study, we used the Nipponbare genome as a reference to map the reads. The alignment results indicated that 70.22–75.39% (67.85–73.17% uniquely matched) of the total reads were mapped to the Nipponbare reference genome and 57.95–63.34% (35.90–38.57% uniquely matched) were mapped to the gene regions (Tables 1 and 2). Meanwhile, there was a significant difference in the percentage of reads mapped to the genome and gene regions, especially for the uniquely mapped reads. These results were similar to those of a previous transcriptome sequencing study of *Sorghum propinquum*, which reported that 72 and 46% of the total reads mapped to the genome and gene regions, respectively, with 68 and 38% of the reads being uniquely matched [31]. This suggested that it might result from reads mapping to intergenic regions and alternative mRNA splicing. Meanwhile, 24.61–29.78% of the DXWR reads remained unmapped, probably due to gaps in the reference genome sequences and diversity between the DXWR and Nipponbare genomes (Table 1). On an average, at least 50% of more than 60% of the mapped genes were covered by uniquely mapped reads, and only approximately 15% of the genes had coverage of 20% or less (Supplementary Figure S2), which indicated that the transcriptome sequences were of high quality.

The article "Effects of drought stress on global gene expression profile in leaf and root samples of Dongxiang wild rice (Oryza rufipogon)" was published in 2017. Journal: Biosci Rep.

**Table 1:** Summary of Illumina transcriptome reads mapped to the reference genome

Reads mapping	Reads number (%)			
	LCK	LD	RCK	RD
Total reads	46784432	48743152	43588908	46684238
Total base pairs	4678443200	4874315200	4358890800	4668423800
Total mapped reads	34881473 (74.56)	36745421 (75.39)	31979139 (73.37)	32781463 (70.22)
Perfect match	25627140 (54.78)	26726941 (54.83)	23267595 (53.38)	23769476 (50.92)
≤3 bp mismatch	9254333 (19.78)	10018480 (20.55)	8711544 (19.99)	9011987 (19.30)
Unique match	34230815 (73.17)	35488839 (72.81)	31136589 (71.43)	31675120 (67.85)
Multiposition match	650658 (1.39)	1256582 (2.58)	842550 (1.93)	1106343 (2.37)
Total unmapped reads	11902959 (25.44)	11997731 (24.61)	11609769 (26.63)	13902775 (29.78)

**Table 2:** Summary of Illumina transcriptome reads mapped to the reference genes

Reads mapping	Reads number (%)			
	LCK	LD	RCK	RD
Total reads	46784432	48743152	43588908	46684238
Total base pairs	4678443200	4874315200	4358890800	4668423800
Total mapped reads	29634341 (63.34)	29171698 (59.85)	26743293 (61.35)	27052687 (57.95)
Perfect match	22232426 (47.52)	21597969 (44.31)	19983467 (45.85)	20078067 (43.01)
≤5 bp mismatch	7401915 (15.82)	7573729 (15.54)	6759826 (15.51)	6974620 (14.94)
Unique match	17816293 (38.08)	17498840 (35.90)	16812042 (38.57)	17068753 (36.56)
Multi-position match	11818048 (25.26)	11672858 (23.95)	9931251 (22.78)	9983934 (21.39)
Total unmapped reads	17150091 (36.66)	19571454 (40.15)	16845615 (38.65)	19631551 (42.05)

### Analysis of DEGs

Based on the number of reads, gene expression levels can be estimated from Illumina sequencing with great accuracy. Putative DEGs from the drought-stressed and control samples (LD compared with LCK and RD compared with RCK) were identified, and 4040 and 7191 transcripts were up- (Supplementary Table S2) and down-regulated (Supplementary Table S3), respectively, in the LD sample, when compared with the LCK sample, whereas 3097 and 3928 transcripts were up- (Supplementary Table S4) and down-regulated (Supplementary Table S5), respectively, in the RD sample, when compared with the RCK sample (Figure 1). Among these DEGs, 1519 and 1459 transcripts were up- (Supplementary Table S6) and down-regulated (Supplementary Table S7), respectively, in both the LD and RD samples, when compared with the control samples (LCK and RCK). Interestingly, 223 transcripts were up-regulated in the LD sample but down-regulated in the RD sample (Supplementary Table S8), and 262 transcripts were down-regulated in the LD sample but up-regulated in the RD sample (Supplementary Table S9).

The article "Effects of drought stress on global gene expression profile in leaf and root samples of Dongxiang wild rice (Oryza rufipogon)" was published in 2017. Journal: Biosci Rep.

**Figure 1:** The number of up- and down-regulated transcripts in the LD and RD compared with the LCK and RCK. LD, leaves with dry treatment; RD, roots with dry treatment; LCK, leaves without dry treatment; RCK, roots without dry treatment.

Quantitative RT-PCR, which was performed to validate the expression data of 30 randomly selected DEGs, yielded results that were highly consistent with those of transcriptome sequencing (*R*^*2*^ =0.9159) (Figure 2). Thus, the DEGs detected in the present study can be considered to have a high accuracy.

**Figure 2:** Comparison of the expression of 30 randomly selected genes using RNA-Seq and qRT-PCR. The gene expression values were transformed to log_2_ scale. The RNA-Seq data log_2_-value (*X*-axis) was plotted against the qRT-PCR log_2_-value (*Y*-axis).

Meanwhile, many DEGs have been previously identified and reported to play roles in the drought stress responses of cultivated rice (Table 3). TFs, for example, have been reported to play essential roles in abiotic stress responses by regulating a large spectrum of downstream stress-responsive genes. Among TF families, the basic leucine zipper (bZIP) family is one of the largest and diverse groups. In plants, bZIP TFs are involved in multiple biological processes that include flower development, seed germination, light signaling, and hormone signaling. In addition, bZIPs are involved in responses to abiotic and biotic stresses [32]. Chen et al. [33] reported that the expression of *OsbZIP16* was dramatically induced under drought conditions and that overexpressing *OsbZIP16* in the *japonica* rice cultivar Zhonghua 11 significantly improved drought resistance at both the seedling and tillering stages. Similarly, Xiang et al. [34] reported that the expression of *OsbZIP23* was strongly induced by a wide spectrum of stresses, including drought, salt, abscisic acid (ABA), and PEG treatments. Furthermore, the overexpression of *OsbZIP23* in the *japonica* rice cultivar Zhonghua 11 significantly improved resistance to drought and high salinity stresses. In the present study, the expression of both *OsbZIP16* and *OsbZIP23* were also significantly induced under drought condition in both leaves and roots, which is consistent with previous reports. In addition to *OsbZIP16* and *OsbZIP23*, the present study also identified six other bZIP TFs, i.e. *OsbZIP4* (*LOC_Os01g36220*), *OsbZIP17* (*LOC_Os02g10140*), *OsbZIP25* (*LOC_Os03g03550*), *OsbZIP48* (*LOC_Os06g39960*), *OsbZIP62* (*LOC_Os07g48660*), and *OsbZIP68* (*LOC_Os08g43090*). Among them, *OsbZIP25, OsbZIP48*, and *OsbZIP68* were up-regulated in both the leaves and roots of drought-stressed plants, whereas *OsbZIP17* and *OsbZIP62* were down-regulated; and *OsbZIP4* was up-regulated in the leaves of drought-stressed plants but down-regulated in the roots.

The article "Effects of drought stress on global gene expression profile in leaf and root samples of Dongxiang wild rice (Oryza rufipogon)" was published in 2017. Journal: Biosci Rep.

**Table 3:** The detected DEGs represented genes that play roles in cultivated rice responses to drought stress

Gene name	Gene ID	Up or down (log_2_ ratio)		References
		LD compared with LCK	RD compared with RCK	
*OsbZIP16*	*LOC_Os02g09830*	Up (3.71)	Up (1.90)	[31]
*OsbZIP23*	*LOC_Os02g52780*	Up (4.06)	Up (3.16)	[32]
*OsDREB2A*	*LOC_Os01g07120*	Up (4.00)	None	[33]
*OsMYB2*	*LOC_Os03g20090*	None	Up (3.40)	[34]
*OsNAC5*	*LOC_Os11g08210*	Up (3.08)	Up (2.50)	[35]
*OsNAC6*	*LOC_Os01g66120*	Up (3.46)	Up (3.21)	[36]
*OsNAC10*	*LOC_Os11g03300*	Up (4.83)	None	[37]
*OsDSS1*	*LOC_Os03g04680*	Down (–2.29)	Down (–1.73)	[38]
*OsWRKY30*	*LOC_Os08g38990*	Up (8.40)	None	[39]
*ZFP182*	*LOC_Os03g60560*	Up (8.63)	Up (6.58)	[40]
*ZFP252*	*LOC_Os12g39400*	Up (3.40)	Up (1.80)	[41]
*OsCPK4*	*LOC_Os02g03410*	Up (1.19)	Up (2.95)	[42]
*DSM2*	*LOC_Os03g03370*	Up (4.86)	Up (3.31)	[43]
*OsABI5*	*LOC_Os01g64000*	Up (5.75)	None	[44]
*OsBIERF3*	*LOC_Os02g43790*	Up (2.72)	Up (3.88)	[45]
*OsTZF1*	*LOC_Os05g10670*	Up (4.10)	None	[46]
*OsDi19-4*	*LOC_Os02g20170*	Up (1.36)	None	[47]
*SNAC1*	*LOC_Os03g60080*	Up (4.61)	Up (5.21)	[48]

Members of another large plant-specific TF superfamily, the NAC TFs, were also identified as DEGs in the present study. Several NAC TFs have previously been demonstrated to function as important regulators of stress responses in cultivated rice. For example, Hu et al. [35] reported that the expression of *SNAC1* was predominantly induced in guard cells by drought stress and that overexpression of *SNAC1* in the *japonica* cultivar Nipponbare significantly enhanced drought resistance in the field, and in the same cultivar, Takasaki et al. [36] reported that the expression of *OsNAC5* was induced by drought, cold, high salinity, ABA, and methyl jasmonic acid, which subsequently enhanced the cultivar’s resistance to drought and high salinity. In addition, Nakashima et al. [37] suggested that the expression of *OsNAC6* could be induced by drought, cold, and high salinity and reported that overexpression of *OsNAC6* improved the Nipponbare cultivar’s resistance to drought and high salinity, and Jeong et al. [38] reported that the expression of *OsNAC10* was induced by drought, high salinity, and ABA and that the overexpression of *OsNAC10* increased the resistance of Nipponbare plants to drought, high salinity, and low temperature. The present study confirmed that drought stress induces the expression *SNAC1, OsNAC5, OsNAC6*, and *OsNAC10* and found that drought stress also affected the expression of two other NAC TFs: *LOC_Os01g60020*, which was up-regulated in both leaves and roots, and *LOC_Os01g50360*, which was up-regulated in leaves but down-regulated in roots. The present study also found that drought stress affects many other TF families, including the MYB, zinc finger, whirly, and WRKY TFs, a finding that is consistent with the opinion that the TFs play important roles in drought resistance in plants [39,40].

The article "Effects of drought stress on global gene expression profile in leaf and root samples of Dongxiang wild rice (Oryza rufipogon)" was published in 2017. Journal: Biosci Rep.

### Functional classification by GO

In the present study, a total of 29350 leaf transcripts in LD compared with LCK and 26656 root transcripts in RD compared with RCK were assigned GO terms. Among the 29350 leaf transcripts, 10360 transcripts were annotated for their cellular component, 9719 were annotated for their molecular function, and 9271 were annotated for their biological process (Figure 3A). Among the 26656 transcripts from the root samples, 9073 transcripts were annotated for their cellular component, 9046 were annotated for their molecular function, and 8537 were annotated for their biological process (Figure 3B). Within the biological process category, cellular and metabolic processes were the most highly represented groups, which suggests that extensive metabolic activities were taking place both in the leaves and roots of the drought-stressed DXWR plants. Meanwhile, within the cellular component category, transcripts that corresponded to cell, cell parts, and cell organelles were the most abundant; and binding and catalytic activities were the most abundant groups within the molecular function category.

**Figure 3:** GO classification of the unigenes from the LD compared with LCK (**A**) and RD compared with RCK (**B**).

We also identified biological process GO terms that were over-represented (*P*<0.05) among the DEGs of LD compared with LCK and RD compared with RCK, respectively (Supplementary Tables S10 and S11). These terms served as indicators of significant biological processes underlying the specific drought-stress responses of leaves and roots. Both sets of transcripts were enriched in GO terms for response to wounding, negative regulation of ABA-mediated signaling pathway, response to inorganic substance, negative regulation of response to alcohol, and response to oxygen-containing compound (Table 4), which suggests that the same biological processes might be involved in the drought responses of both the tissues.

The article "Effects of drought stress on global gene expression profile in leaf and root samples of Dongxiang wild rice (Oryza rufipogon)" was published in 2017. Journal: Biosci Rep.

**Table 4:** The significant GO terms of DEGs for the biological process category both in the LD compared with LCK and RD compared with RCK

GO term	GO term annotation
GO:0009611	Response to wounding
GO:0009788	Negative regulation of ABA-mediated signaling pathway
GO:0010035	Response to inorganic substance
GO:1901420	Negative regulation of response to alcohol
GO:1901700	Response to oxygen-containing compound

Meanwhile, in regard to the over-representation of cellular component terms (*P*<0.05) among the LD, LCK, RD, and RCK samples (Supplementary Tables S12–S15, respectively), we found chloroplast thylakoid, chloroplast thylakoid membrane, thylakoid, plastid thylakoid, thylakoid membrane, thylakoid part, and plastid thylakoid membrane were enriched in both sets of transcripts from each tissue (Supplementary Table S16). This is consistent with the opinion that the thylakoid is one of the most important cellular components for the normal growth and development of plants and that it is also involved in drought resistance [41,42]. Tian et al. [43] reported that the stay-green wheat mutant *tasg1* exhibited greater functional stability of its thylakoid membrane proteins than the wild-type parent and that *tasg1* mutants maintained higher Hill activity, actual efficiency (*Φ*_PSII_), maximal photochemical efficiency of PSII (*F*_v_/*F*_m_), and Ca^2+^-ATPase and Mg^2+^-ATPase activities under drought stress, thus conferring improved drought resistance.

For the molecular function category, endopeptidase inhibitor activity, endopeptidase regulator activity, and serine-type endopeptidase inhibitor activity were enriched in both tissues (Supplementary Table S17). This suggested that the expression of some stress-responsive genes might be regulated by post-translational modification. In addition, iron ion binding and electron carrier activity were also enriched in both tissues, which is consistent with recent studies and suggests that these DEGs play key roles in mitigating the harmful effects of drought stress [44,45].

The article "Effects of drought stress on global gene expression profile in leaf and root samples of Dongxiang wild rice (Oryza rufipogon)" was published in 2017. Journal: Biosci Rep.

### KEGG pathway mapping

The KEGG pathway based analysis indicated that 7056 of the 11231 leaf DEGs and 4115 of the 7025 root DEGs could be classified into 20 functional categories and 128 and 126 subcategories, respectively. Furthermore, the over-represented KEGG orthology (KO) terms (*Q*-value <0.05) could be classified into 10 and 12 categories, respectively (Figure 4), and the most common KO terms represented by both the leaf and root DEGs included global map, translation, lipid metabolism, signal transduction, biosynthesis of other secondary metabolites, metabolism of terpenoids and polyketides, carbohydrate metabolism, and amino acid metabolism.

**Figure 4:** KEGG pathway assignments in the LD compared with LCK (**A**) and RD compared with RCK (**B**). The represented categories (*Q*-value ≤0.05) and the number of transcripts predicted to belong to each category are shown.

The over-represented KO terms for the leaf and root DEGs were further classified into 23 and 28 subcategories, respectively (Supplementary Tables S18 and S19). Among these subcategories, 11 subcategories were over-represented among both the leaf and root DEGs (Supplementary Figure S3), including tryptophan metabolism; RNA transport; plant hormone signal transduction; mRNA surveillance pathway; limonene and pinene degradation; isoflavonoid biosynthesis; flavone and flavonol biosynthesis; cutin, suberine, and wax biosynthesis; biosynthesis of secondary metabolites; benzoxazinoid biosynthesis and stilbenoid, and diarylheptanoid and gingerol biosynthesis. Among these terms, RNA transport and the mRNA surveillance pathway are related to transcription. Thus, the pathways might modulate the regulation of drought-induced gene expression.

Furthermore, 17 KO terms were exclusively among the root DEGs and 12 KO terms were exclusively enriched among the leaf DEGs. This finding suggests that there could be considerable differences in the biochemical and physiological processes involved in the drought responses of leaves and roots, and these annotations provide a valuable resource for investigating the specific processes, functions, and pathways involved in such differences.

### DEGs and previously identified drought resistance related QTL intervals

Until now, only 12 drought resistance-related QTLs had been identified in DXWR [12]. These were located on chromosomes 2, 4, 5, 6, 8, 9, and 12; and among the 12 QTLs, *qSDT2-1* and *qSDT12-2* had been identified as the two most significant QTLs for drought resistance, explaining up to 7 and 14% of the phenotypic variance and possessing positive additive effects of 1.2 and 1.38, respectively [12]. Furthermore, *qSDT2-1* was mapped within 15.9 cM on chromosome 2, and *qSDT12-2* was mapped within 6.7 cM on chromosome 12 [12].

The article "Effects of drought stress on global gene expression profile in leaf and root samples of Dongxiang wild rice (Oryza rufipogon)" was published in 2017. Journal: Biosci Rep.

In the present study, a total of 146 and 81 DEGs were co-localized within the *qSDT2-1* and *qSDT12-2* intervals, respectively (Supplementary Table S20). To identify the most interesting candidate genes, the DEGs with absolute log_2_RPKM ratio values of ≥2 (in at least one tissue) were isolated for further analysis. This screening reduced the total number of DEGs in the *qSDT2-1* interval to 71, which included 42 leaf DEGs (16 up-regulated and 26 down-regulated), 22 root DEGs (8 up-regulated and 14 down-regulated), and 7 DEGs that were differentially expressed in both leaves and roots (5 up-regulated and 2 down-regulated; Supplementary Table S20). Similarly, screening reduced the total number of DEGs in the *qSDT12-2* interval to 43, which included 24 leaf DEGs (5 up-regulated and 19 down-regulated), 15 root DEGs (5 up-regulated and 10 down-regulated), 3 DEGs that were differentially expressed in both leaves and roots (2 up-regulated and 1 down-regulated), and 1 DEG that exhibited a contrasting expression pattern, being up-regulated in leaves and down-regulated in roots (Supplementary Table S20).

Many of these DEGs are involved in the resistance of plants to abiotic stress. For example, Cui et al. [46] reported that *OsSGL* (*LOC_Os02g04130*), which encodes a DUF1645 domain containing protein, can be induced by multiple stresses, and the over- or hetero-expression of *OsSGL* have been reported to significantly improve the drought resistance of transgenic rice and *Arabidopsis thaliana*, respectively. Here, in the present study, the expression of *LOC_Os02g04130* was also significantly up-regulated by drought stress, in both leaves and roots. Previous studies have also suggested that the genes encoding 9-*cis*-epoxycarotenoid dioxygenase play important roles in regulating endogenous ABA levels and contributes to drought stress resistance [47–49]. Indeed, the present study observed that the expression of *LOC_Os12g42280*, which putatively encodes 9-*cis*-epoxycarotenoid dioxygenase 1, was up-regulated in both leaves and roots under drought stress. Furthermore, the ubiquitin system plays a key role in plant biology by interfering with key components of important pathways, including those associated with abiotic stress, immunity, and hormonal signaling [50]. The present study also found that *LOC_Os02g06640*, which putatively encodes a ubiquitin family protein, was significantly up-regulated in leaves under drought stress.

In addition, protein kinases, which constitute one of the largest gene families in plants, play critical roles in the regulation of cellular pathways, signal transduction, and plant development, and many protein kinases are involved in the drought-stress responses [51]. For example, overexpression of an *Arabidopsis* cysteine-rich receptor-like protein kinase, *CRK5*, was reported to enhance ABA sensitivity and confer drought resistance [52]. In the present study, eight protein kinase-encoding genes were significantly affected by drought stress: *LOC_Os02g04240, LOC_Os02g05820, LOC_Os02g06930, LOC_Os02g08530, LOC_Os12g41090, LOC_Os12g41510, LOC_Os12g42040*, and *LOC_Os12g42070*. Transposons and retrotransposon, which are also important upstream regulators of plant drought stress responses [53,54], were identified by the present study, as well (*LOC_Os02g04150, LOC_Os02g04540, LOC_Os02g05550, LOC_Os02g07270, LOC_Os02g07370, LOC_Os02g07380, LOC_Os02g07400*, and *LOC_Os02g07570*), as were various other types of TFs, including zinc finger TFs (*LOC_Os02g07930, LOC_Os02g08510*, and *LOC_Os12g42970*), bZip TFs (*LOC_Os02g05640* and *LOC_Os12g40920*), and MYB TFs (*LOC_Os02g04640* and *LOC_Os02g07170*). These co-localized and drought-affected DEGs identified in the present study provide a basis for future studies aiming to elucidate the molecular mechanisms of drought resistance in rice.

The article "Effects of drought stress on global gene expression profile in leaf and root samples of Dongxiang wild rice (Oryza rufipogon)" was published in 2017. Journal: Biosci Rep.

## Conclusion

The present study investigated the superior drought resistance of DXWR, which is highly valuable for genetic research and the breeding of drought resistance in rice. This work presented an original transcriptome analysis of drought-stressed DXWR leaf and root tissues. A large number of DEGs were identified; and several key pathways, including those for RNA transport, mRNA surveillance, secondary metabolite biosynthesis, and plant hormone signal transduction, and various processes, including endopeptidase inhibitor activity, serine-type endopeptidase inhibitor activity, iron ion binding, and electron carrier activity were identified as involved in drought resistance. By combining the DEGs identified in the present study with previously identified drought-resistance QTLs from DXWR, the most interesting candidate genes were identified, including various TFs, protein kinases, and other functional proteins. These findings will be useful in future studies of molecular adaptations to drought stress and will facilitate the genetic manipulation of rice to improve its drought resistance.

## Abbreviations

ABA: abscisic acid
bZIP: basic leucine zipper
DEG: differentially expressed gene
DXWR: Dongxiang wild rice
GO: gene ontology
IRRI: International Rice Research Institute
KEGG: Kyoto encyclopedia of genes and genomes
KO: KEGG orthology
LCK: leaves without dry treatment
LD: leaves with dry treatment
qRT-PCR: quantitative real-time PCR
QTL: quantitative trait loci
RCK: roots without dry treatment
RD: roots with dry treatment
RPKM: reads per kilobase per million reads
TF: transcription factor
COG: Clusters of Orthologous Groups

The article "Effects of drought stress on global gene expression profile in leaf and root samples of Dongxiang wild rice (Oryza rufipogon)" was published in 2017. Journal: Biosci Rep.

## References

[1] JaleelC.A., ManivannanP., WahidA., FarooqM., Al-JuburiH.J., SomasundaramR. (2009) Drought stress in plants: a review on morphological characteristics and pigments composition. Int. J. Agric. Biol. 11, 100–105

[2] KrannichC.T., MaletzkiL., KurowskyC. and HornR. (2015) Network candidate genes in breeding for drought tolerant crops. Int. J. Mol. Sci. 16, 16378–164002619326910.3390/ijms160716378PMC4519955

[3] ZhaoK., TungC.W., EizengaG.C., WrightM.H., AliM.L., PriceA.H. (2011) Genome-wide association mapping reveals a rich genetic architecture of complex traits in *Oryza sativa*. Nat. Commun. 2, 4672191510910.1038/ncomms1467PMC3195253

[4] FukaoT. and XiongL.Z. (2013) Genetic mechanisms conferring adaptation to submergence and drought in rice: simple or complex? Curr. Opin. Plant Biol. 16, 196–2042345378010.1016/j.pbi.2013.02.003

[5] HadiartoT. and TranL.S. (2011) Progress studies of drought-responsive genes in rice. Plant Cell Rep. 30, 297–3102113243110.1007/s00299-010-0956-z

[6] DegenkolbeT., DoP.T., ZutherE., RepsilberD., WaltherD., HinchaD.K. (2009) Expression profiling of rice cultivars differing in their tolerance to long-term drought stress. Plant Mol. Biol. 69, 133–1531893197610.1007/s11103-008-9412-7PMC2709230

[7] WangD., PanY.J., ZhaoX.Q., ZhuL.H., FuB.Y. and LiZ.K. (2011) Genome-wide temporal-spatial gene expression profiling of drought responsiveness in rice. BMC Genomics 12, 1492140611610.1186/1471-2164-12-149PMC3070656

[8] LenkaS.K., KatiyarA., ChinnusamyV. and BansalK.C. (2011) Comparative analysis of drought-responsive transcriptome in *Indica* rice genotypes with contrasting drought tolerance. Plant Biotechnol. J. 9, 315–3272080992810.1111/j.1467-7652.2010.00560.x

[9] XieJ.K., AgramaH.A., KongD., ZhuangJ., HuB.L., WanY. (2010) Genetic diversity associated with conservation of endangered Dongxiang wild rice (*Oryza rufipogon*). Genet. Resour. Crop Ev. 57, 597–609

[10] ZhangF.T., CuiF.L., ZhangL.X., WenX.F., LuoX.D., ZhouY. (2014) Development and identification of a introgression line with strong drought resistance at seedling stage derived from *Oryza sativa* L. mating with *Oryza rufipogon* Griff. Euphytica 200, 1–7

[11] ZhangF.T., LuoX.D., ZhouY. and XieJ.K. (2016) Genome-wide identification of conserved microRNA and their response to drought stress in Dongxiang wild rice (*Oryza rufipogon* Griff.). Biotechnol. Lett. 38, 711–7212666713310.1007/s10529-015-2012-0

[12] ZhangX., ZhouS.X., FuY.C., SuZ., WangX.K. and SunC.Q. (2006) Identification of a drought tolerant introgression line derived from Dongxiang common wild rice (*O. rufipogon* Griff.). Plant Mol. Biol. 62, 247–2591684547910.1007/s11103-006-9018-x

The article "Effects of drought stress on global gene expression profile in leaf and root samples of Dongxiang wild rice (Oryza rufipogon)" was published in 2017. Journal: Biosci Rep.

[13] MofattoL.S., CarneiroF.A., VieiraN.G., DuarteK.E., VidalR.O., AlekcevetchJ.C. (2016) Identification of candidate genes for drought tolerance in coffee by high-throughput sequencing in the shoot apex of different *Coffea arabica* cultivars. BMC Plant Biol. 16, 942709527610.1186/s12870-016-0777-5PMC4837521

[14] HuW., XiaZ.Q., YanY., DingZ.H., TieW.W., WangL.Z. (2015) Genome-wide gene phylogeny of CIPK family in cassava and expression analysis of partial drought-induced genes. Front. Plant Sci. 6, 9142657916110.3389/fpls.2015.00914PMC4626571

[15] FracassoA., TrindadeL.M. and AmaducciS. (2016) Drought stress tolerance strategies revealed by RNA-Seq in two sorghum genotypes with contrasting WUE. BMC Plant Biol. 16, 1152720897710.1186/s12870-016-0800-xPMC4875703

[16] BrasileiroA.C., MorganteC.V., AraujoA.C., Leal-BertioliS.C., SilvaA.K., MartinsA.C. (2015) Transcriptome profiling of wild *Arachis* from water-limited environments uncovers drought tolerance candidate genes. Plant Mol. Biol. Report 33, 1876–18922675280710.1007/s11105-015-0882-xPMC4695501

[17] XuJ., YuanY.B., XuY.B., ZhangG.Y., GuoX.S., WuF.K. (2014) Identification of candidate genes for drought tolerance by whole-genome resequencing in maize. BMC Plant Biol. 14, 832468480510.1186/1471-2229-14-83PMC4021222

[18] FengH.M., YanM., FanX.R., LiB.Z., ShenQ.R., MillerA.J. (2011) Spatial expression and regulation of rice high-affinity nitrate transporters by nitrogen and carbon status. J. Exp. Bot. 62, 2319–23322122078110.1093/jxb/erq403

[19] ZhouY., YangP., CuiF.L., ZhangF.T., LuoX.D. and XieJ.K. (2016) Transcriptome analysis of salt stress responsiveness in the seedlings of Dongxiang wild rice (*Oryza rufipogon* Griff.). PLoS ONE 11, e01462422675240810.1371/journal.pone.0146242PMC4709063

[20] LiB. and DeweyC.N. (2011) RSEM: accurate transcript quantification from RNA-Seq data with or without a reference genome. BMC Bioinformatics 12, 3232181604010.1186/1471-2105-12-323PMC3163565

[21] TrapnellC., PachterL. and SalzbergS.L. (2009) TopHat: discovering splice junctions with RNA-Seq. Bioinformatics 25, 1105–11111928944510.1093/bioinformatics/btp120PMC2672628

[22] TrapnellC., WilliamsB.A., PerteaG., MortazaviA., KwanG., van BarenM.J. (2010) Transcript assembly and quantification by RNA-Seq reveals unannotated transcripts and isoform switching during cell differentiation. Nat. Biotechnol. 28, 511–5152043646410.1038/nbt.1621PMC3146043

[23] TianX.J., LongY., WangJ., ZhangJ.W., WangY.Y., LiW.M. (2015) *De novo* transcriptome assembly of common wild rice (*Oryza rufipogon* Griff.) and discovery of drought-response genes in root tissue based on transcriptomic data. PLoS ONE 10, e01314552613413810.1371/journal.pone.0131455PMC4489613

The article "Effects of drought stress on global gene expression profile in leaf and root samples of Dongxiang wild rice (Oryza rufipogon)" was published in 2017. Journal: Biosci Rep.

[24] ConesaA. and GötzS. (2008) Blast2GO: a comprehensive suite for functional analysis in plant genomics. Int. J. Plant Genomics 2008, 6198321848357210.1155/2008/619832PMC2375974

[25] MortazaviA., WilliamsB.A., McCueK., SchaefferL. and WoldB. (2008) Mapping and quantifying mammalian transcriptomes by RNA-Seq. Nat. Methods 5, 621–6281851604510.1038/nmeth.1226PMC13303166

[26] BenjaminiY. and YekutieliD. (2001) The control of the false discovery rate in multiple testing under dependency. Ann. Stat. 29, 1165–1188

[27] ZhangF.T., LuoX.D., HuB.L., WanY. and XieJ.K. (2013) *YGL138*(t), encoding a putative signal recognition particle 54 kDa protein, is involved in chloroplast development of rice. Rice 6, 72428053710.1186/1939-8433-6-7PMC4883693

[28] OkaH.I. (2012) Origin of Cultivated Rice, Elsevier, Philadelphia

[29] KawaharaY., de la BastideM., HamiltonJ.P., KanamoriH., McCombieW.R., OuyangS. (2013) Improvement of the *Oryza sativa* Nipponbare reference genome using next generation sequence and optical map data. Rice 6, 42428037410.1186/1939-8433-6-4PMC5395016

[30] ZhangF.T., XuT., MaoL.Y., YanS.Y., ChenX.W., WuZ.F. (2016) Genome-wide analysis of Dongxiang wild rice (*Oryza rufipogon* Griff.) to investigate lost/acquired genes during rice domestication. BMC Plant Biol. 16, 1032711839410.1186/s12870-016-0788-2PMC4845489

[31] ZhangT., ZhaoX.Q., WangW.S., HuangL.Y., LiuX.Y., ZongY. (2014) Deep transcriptome sequencing of rhizome and aerial-shoot in *Sorghum propinquum*. Plant Mol. Biol. 84, 315–3272410486210.1007/s11103-013-0135-z

[32] SornarajP., LuangS., LopatoS. and HrmovaM. (2016) Basic leucine zipper (bZIP) transcription factors involved in abiotic stresses: a molecular model of a wheat bZIP factor and implications of its structure in function. Biochim. Biophys. Acta 1860, 46–562649372310.1016/j.bbagen.2015.10.014

[33] ChenH., ChenW., ZhouJ.L., HeH., ChenL.B., ChenH.D. (2012) Basic leucine zipper transcription factor OsbZIP16 positively regulates drought resistance in rice. Plant Sci. 193–194, 8–1710.1016/j.plantsci.2012.05.00322794914

[34] XiangY., TangN., DuH., YeH.Y. and XiongL.Z. (2008) Characterization of *OsbZIP23* as a key player of the basic leucine zipper transcription factor family for conferring abscisic acid sensitivity and salinity and drought tolerance in rice. Plant Physiol. 148, 1938–19521893114310.1104/pp.108.128199PMC2593664

[35] HuH.H., DaiM.Q., YaoJ.L., XiaoB.Z., LiX.H., ZhangQ.F. (2006) Overexpressing a NAM, ATAF, and CUC (NAC) transcription factor enhances drought resistance and salt tolerance in rice. Proc. Natl. Acad. Sci. U.S.A. 103, 12987–129921692411710.1073/pnas.0604882103PMC1559740

The article "Effects of drought stress on global gene expression profile in leaf and root samples of Dongxiang wild rice (Oryza rufipogon)" was published in 2017. Journal: Biosci Rep.

[36] TakasakiH., MaruyamaK., KidokoroS., ItoY., FujitaY., ShinozakiK. (2010) The abiotic stress-responsive NAC-type transcription factor *OsNAC5* regulates stress-inducible genes and stress tolerance in rice. Mol. Genet. Genomics 284, 173–1832063203410.1007/s00438-010-0557-0

[37] NakashimaK., TranL.S., Van NguyenD., FujitaM., MaruyamaK., TodakaD. (2007) Functional analysis of a NAC-type transcription factor *OsNAC6* involved in abiotic and biotic stress-responsive gene expression in rice. Plant J. 51, 617–6301758730510.1111/j.1365-313X.2007.03168.x

[38] JeongJ.S., KimY.S., BaekK.H., JungH., HaS.H., Do ChoiY. (2010) Root-specific expression of *OsNAC10* improves drought tolerance and grain yield in rice under field drought conditions. Plant Physiol. 153, 185–1972033540110.1104/pp.110.154773PMC2862432

[39] JoshiR., WaniS.H., SinghB., BohraA., DarZ.A., LoneA.A. (2016) Transcription factors and plants response to drought stress: current understanding and future directions. Front. Plant Sci. 7, 10292747151310.3389/fpls.2016.01029PMC4943945

[40] GahlautV., JaiswalV., KumarA. and GuptaP.K. (2016) Transcription factors involved in drought tolerance and their possible role in developing drought tolerant cultivars with emphasis on wheat (*Triticum aestivum* L.). Theor. Appl. Genet. 129, 2019–20422773871410.1007/s00122-016-2794-z

[41] ChenY.E., LiuW.J., SuY.Q., CuiJ.M., ZhangZ.W., YuanM. (2016) Different response of photosystem II to short and long-term drought stress in *Arabidopsis thaliana*. Physiol. Plantarum 158, 225–23510.1111/ppl.1243826918860

[42] WangS. and BlumwaldE. (2014) Stress-induced chloroplast degradation in *Arabidopsis* is regulated via a process independent of autophagy and senescence-associated vacuoles. Plant Cell 26, 4875–48882553818610.1105/tpc.114.133116PMC4311210

[43] TianF., GongJ., ZhangJ., ZhangM., WangG., LiA. (2013) Enhanced stability of thylakoid membrane proteins and antioxidant competence contribute to drought stress resistance in the *tasg1* wheat stay-green mutant. J. Exp. Bot. 64, 1509–15202337837610.1093/jxb/ert004PMC3617820

[44] WuH.M., ZhengY., LiuJ., ZhangH.T. and ChenH.P. (2016) Heme oxygenase-1 delays gibberellin-induced programmed cell death of rice aleurone layers subjected to drought stress by interacting with nitric oxide. Front. Plant Sci. 6, 12672683476910.3389/fpls.2015.01267PMC4717306

[45] PrinceS.J., JoshiT., MutavaR.N., SyedN., Joao Vitor MdosS., PatilG. (2015) Comparative analysis of the drought-responsive transcriptome in soybean lines contrasting for canopy wilting. Plant Sci 240, 65–782647518810.1016/j.plantsci.2015.08.017

The article "Effects of drought stress on global gene expression profile in leaf and root samples of Dongxiang wild rice (Oryza rufipogon)" was published in 2017. Journal: Biosci Rep.

[46] CuiY.C., WangM.L., ZhouH.N., LiM.J., HuangL.F., YinX.M. (2016) *OsSGL*, a novel DUF1645 domain-containing protein, confers enhanced drought tolerance in transgenic rice and *Arabidopsis*. Front. Plant Sci. 7, 20012808301310.3389/fpls.2016.02001PMC5186801

[47] EspasandinF.D., MaialeS.J., CalzadillaP., RuizO.A. and SansberroP.A. (2014) Transcriptional regulation of 9-*cis*-epoxycarotenoid dioxygenase (NCED) gene by putrescine accumulation positively modulates ABA synthesis and drought tolerance in *Lotus tenuis* plants. Plant Physiol. Biochem. 76, 29–352444832210.1016/j.plaphy.2013.12.018

[48] XianL., SunP., HuS., WuJ. and LiuJ.H. (2014) Molecular cloning and characterization of *CrNCED1*, a gene encoding 9-*cis*-epoxycarotenoid dioxygenase in *Citrus reshni*, with functions in tolerance to multiple abiotic stresses. Planta 239, 61–772406830010.1007/s00425-013-1963-4

[49] EndoA., SawadaY., TakahashiH., OkamotoM., IkegamiK., KoiwaiH. (2008) Drought induction of *Arabidopsis* 9-*cis*-epoxycarotenoid dioxygenase occurs in vascular parenchyma cells. Plant Physiol. 147, 1984–19931855068710.1104/pp.108.116632PMC2492653

[50] SharmaB., JoshiD., YadavP.K., GuptaA.K. and BhattT.K. (2016) Role of ubiquitin-mediated degradation system in plant biology. Front. Plant Sci. 7, 8062737566010.3389/fpls.2016.00806PMC4897311

[51] YeY.Y., DingY.F., JiangQ., WangF.J., SunJ.W. and ZhuC. (2017) The role of receptor-like protein kinases (RLKs) in abiotic stress response in plants. Plant Cell Rep. 36, 235–2422793337910.1007/s00299-016-2084-x

[52] LuK., LiangS., WuZ., BiC., YuY.T., WangX.F. (2016) Overexpression of an *Arabidopsis* cysteine-rich receptor-like protein kinase, CRK5, enhances abscisic acid sensitivity and confers drought tolerance. J. Exp. Bot. 67, 5009–50272740678410.1093/jxb/erw266PMC5014153

[53] PiacentiniL., FantiL., SpecchiaV., BozzettiM.P., BerlocoM., PalumboG. (2014) Transposons, environmental changes, and heritable induced phenotypic variability. Chromosoma 123, 345–3542475278310.1007/s00412-014-0464-yPMC4107273

[54] ForestanC., AieseC.R., FarinatiS., LunardonA., SanseverinoW. and VarottoS. (2016) Stress-induced and epigenetic-mediated maize transcriptome regulation study by means of transcriptome reannotation and differential expression analysis. Sci. Rep. 6, 304462746113910.1038/srep30446PMC4962059

